# LncRNA-XIST interacts with *miR-29c* to modulate the chemoresistance of glioma cell to TMZ through DNA mismatch repair pathway

**DOI:** 10.1042/BSR20170696

**Published:** 2017-09-07

**Authors:** Peng Du, Haiting Zhao, Renjun Peng, Qing Liu, Jian Yuan, Gang Peng, Yiwei Liao

**Affiliations:** 1 Department of Neurosurgery, The Second Affiliated Hospital, Xinjiang Medical University, Urumqi 830063, P.R. China; 2 Department of Neurology, Xiangya Hospital, The Central South University (CSU), Changsha 410008, P.R. China; 3 Department of Neurosurgery, Xiangya Hospital, The Central South University (CSU), Changsha 410008, P.R. China

**Keywords:** chemoresistance, glioma, lncRNA-XIST, miR-29c, Temozolomide (TMZ)

## Abstract

Temozolomide (TMZ) is the most commonly used alkylating agent in glioma chemotherapy. However, growing resistance to TMZ remains a major challenge for clinicians. Recent evidence emphasizes the key regulatory roles of non-coding RNAs (lncRNAs and miRNAs) in tumor biology, including the chemoresistance of cancers. However, little is known about the role and regulation mechanisms of lncRNA cancer X-inactive specific transcripts (XIST) in glioma tumorigenesis and chemotherapy resistance. In the present study, higher XIST expression was observed in glioma tissues and cell lines, which was related to poorer clinicopathologic features and shorter survival time. XIST knockdown alone was sufficient to inhibit glioma cell proliferation and to amplify TMZ-induced cell proliferation inhibition. Moreover, XIST knockdown can sensitize TMZ-resistant glioma cells to TMZ. XIST can inhibit *miR-29c* expression by directly targetting TMZ-resistant glioma cells. DNA repair protein O^6^-methylguanine-DNA methytransferase (MGMT) plays a key role in TMZ resistance; transcription factor specificity protein 1 (SP1), a regulator of DNA mismatch repair (MMR) key protein MSH6, has been reported to be up-regulated in TMZ-resistant glioma cell lines. In the present study, we show that XIST/*miR-29c* coregulates SP1 and MGMT expression in TMZ-resistant glioma cell lines. Our data suggest that XIST can amplify the chemoresistance of glioma cell lines to TMZ through directly targetting *miR-29c* via SP1 and MGMT. XIST/*miR-29c* may be a potential therapeutic target for glioma treatment.

## Introduction

As the most common brain cancer, glioma accounts for >60% of primary brain tumors in adults [1,2]. Surgery followed by radiotherapy, with temozolomide (TMZ) adjuvant chemotherapy, is the standard treatment for glioma; however, the prognosis remains poor due to the growing resistance to TMZ [1,3]. The pathogenesis of glioma is largely unknown, although it has been shown that genetic changes in many genes are associated with the development of glioma [4–6]. Therefore, investigating the pathogenesis of glioma and the mechanism of chemoresistance acquisition are critically important for the diagnosis and treatment of this fatal disease.

In recent years, emerging evidence has regarded non-coding RNAs, including lncRNAs and miRNAs as major regulators of normal development and diseases, including cancer [7–9]. Under different circumstances, lncRNAs and miRNAs can play a role in tumorigenesis, tumor inhibition, or both [10–12]. The lncRNA X inactive specific transcript (XIST) has been found to be up-regulated and acts as a carcinogen in glioblastoma [13], ovarian cancer [14], and non-small-cell lung cancer [15]. In addition, its role in cancer resistance to chemotherapy has also been reported [16,17]; however, little is known about its expression pattern, biological function and potential mechanism of glioma progression, and the chemoresistance of glioma to TMZ. In addition to XIST, the role of *miR-29c* in cancers has been extensively studied. Through inhibiting cancer cell proliferation, invasion, and/or migration, *miR-29c* acts as a tumor suppressor in gastric cancer [18], pancreatic cancer [19], colorectal cancer [20], and so on. More importantly, *miR-29c* has been reported to regulate the radioresistance of cancer cells in lung cancer [21].

It has been recently discovered that the interactions between lncRNAs and miRNAs affect post-transcriptional regulation by inhibiting the available miRNA activity. According to previous studies, lncRNA can act as a specific ‘sponge’ for miRNA to reduce their regulation of mRNA [22]. Whether XIST can interact with *miR-29c* to affect glioma cell proliferation and its chemoresistance to TMZ remain to be uncovered.

In the present study, the expression levels of XIST in glioma tissues and the peritumoral brain edema (PTBE) tissues, the relationship between XIST expression and the clinical features in patients with glioma, and the effects of XIST on glioma cell proliferation and chemoresistance to TMZ were evaluated. Further, we revealed that the interaction between XIST and *miR-29c* regulates the chemosensitivity to TMZ-based chemotherapy through specificity protein 1 (SP1) and O^6^-methylguanine-DNA methytransferase (MGMT). Our findings provide a novel understanding of the function of XIST/*miR-29c*/SP1/MGMT in the sensitivity of glioma to chemotherapy and the mechanism involved.

## Materials and methods

### Cell lines, tissues, and transfection

With the approval of the Ethical Committee of Xiangya Hospital, the Central South University (CSU), we collected 69 paired glioma tissues as well as the PTBE tissues. All the samples were obtained from patients who underwent surgical resection at Xiangya Hospital, CSU (Changsha, China). All the tissue samples were snap-frozen and stored at –80°C in liquid nitrogen. The clinical features of patients are listed in Table 1. Univariate and multivariate analyses of factors related to oversurvival using the COX proportional hazard model is listed in Table 2.

**Table 1:** Correlation of the expression of XIST with clinicopathologic features

Characteristics	*n*	Relative XIST expression		*P*-value
		High	Low	
***Age***				0.921
<45 years	28	14	14	
≥45 years	41	21	20	
***Gender***				0.537
Female	31	17	14	
Male	38	18	20	
***Tumor size***				0.003
<5 cm	32	10	22	
≥5 cm	37	25	12	
***PTBE***				0.116
≥1 cm	36	15	21	
<1 cm	33	20	13	
***WHO stage***				<0.001
I + II	33	6	27	
III + IV	36	29	7	

**Table 2:** Univariate and multivariate analyses for factors related to oversurvival using the COX proportional hazard model

Characteristics		Univariate analysis		Multivariate analysis	
		HR (95% CI)	*P*-value	HR (95% CI)	*P*-value
Age	<45 compared with ≥45	0.747 (0.422–1.324)	0.318	N.A.	
Gender	female compared with male	0.908 (0.521–1.583)	0.735	N.A.	
Tumor size	≥5 cm compared with <5 cm	0.825 (0.472–1.444)	0.502	N.A.	
PTBE	≥1 cm compared with <1 cm	1.030 (0.591–1.795)	0.917	N.A.	
WHO stage	I + II compared with III + IV	0.428 (0.242–0.756)	0.004	0.571 (0.306–1.067)	0.079
XIST expression	high compared with low	2.560 (1.438–4.557)	0.001	2.037 (1.083–3.831)	0.027

N.A., not applicable.

Human glioma cell lines: U251, U373, LN229, U118, and LN229, as well as a normal cell line, normal human astrocytes (NHA) were obtained from the American Type Culture Collection (ATCC, U.S.A.), cultured in 10% FBS (Gibco, U.S.A.) supplemented RPMI-1640 medium (Invitrogen, U.S.A.) at 37 °C with 5% v/v CO_2_.

LN229 and U251 glioma cells, normally sensitive to TMZ, were cultured in incremental concentrations of TMZ up to 400 µM over several weeks in our laboratory with stepwise selection and the subculture of resistant clones as described by Zhang et al. [23].

*MiR-29c* mimic or *miR-29c* inhibitor (GenePharma, China) was transfected into the indicated target cells to achieve *miR-29c* overexpression or *miR-29c* inhibition by using Lipofectamine 2000 (Invitrogen). SiRNA-XIST was used to achieve knockdown of XIST (GeneCopoeia, China).

### Real-time PCR

TRIzol reagent (Invitrogen) was used for total RNA extraction following the manufacturer’s instructions. By using miRNA-specific primer, total RNA was reverse transcribed and the miScript Reverse Transcription Kit (Qiagen, Germany) was used for *miR-29c* qRT-PCR. The SYBR Green PCR Master Mix (Qiagen) was used following the manufacturer’s instructions. The *C*_t_ method was used to evaluate the relative expression and normalized to U6 expression. The First-strand cDNA Synthesis Kit (Promega, U.S.A.) was used to perform the reverse transcription to determine XIST expression following the manufacturer’s instructions. The expression of *GAPDH* mRNA was regarded as an internal control.

### Western blotting

RIPA buffer (Cell Signaling Technology, U.S.A.) was used to homogenize the cells. The expression of SP1 and MGMT in glioma cells was detected by performing immunoblotting. Cells were lysed, cultured, or transfected in 1% PMSF supplemented RIPA buffer. Protein was loaded on to SDS/PAGE minigel, and then transferred on to PVDF membrane. The blots were probed with the following antibodies: anti-SP1 (Cat# EPR6662 (B), Abcam, U.S.A.), anti-MGMT (Cat# EPR4397, Abcam, U.S.A.), and anti-GAPDH (Cat# 6C5, Abcam, U.S.A.) at 4°C overnight, and incubated with HRP–conjugated secondary antibody (1:5000). Signals were visualized using ECL Substrates (Millipore, U.S.A.). The protein expression was normalized to endogenous GAPDH.

### Luciferase activity

LN229 cells were cultured overnight after being seeded into a 24-well plate, cotransfected with the wt-XIST or mut-XIST reporter gene plasmid containing a 5-bp mutation in the predicted binding site of *miR-29c* and *miR-29c* mimics or *miR-29c* inhibitor. Forty-eight hours after transfection, Dual Luciferase Reporter Assay System (Promega, U.S.A.) was used to perform the luciferase assays.

### RNA immunoprecipitation

LN229/TMZ and U251/TMZ cell lysates were used for RNA immunoprecipitation (RIP). The Imprint RNA Immunoprecipitation Kit (Sigma, U.S.A.) was used in RIP with the AGO2 antibody (ab32381, Abcam, U.S.A.), which is a key component of the miRNA-containing RNA-induced silencing complex (RISC). AGO2 was used as positive controls and IgG as the negative controls. The levels of XIST and *miR-29c* in the precipitates were determined using real-time PCR.

### MTT assay

Twenty four hours after seeding into 96-well plates (5000 cells per well), cells were transfected with siRNA-XIST. Twenty four hours post-transfection, cells were exposed to TMZ (0, 7.5, 15, 30, 60, 120, 240, and 480 μM) for another 24 h. Then, 20 μl MTT (at a concentration of 5 mg/ml; Sigma–Aldrich) was added, and the cells were incubated for an additional 4 h in a humidified incubator. DMSO (200 μl) was added after the supernatant discarded to dissolve the formazan. OD_490 nm_ value was measured. The viability of the untreated cells (control) was defined as 100%, and the viability of cells from all other groups was calculated separately from that of the control group.

### BrdU incorporation assay

By measuring 5-Bromo-2-deoxyuridine (BrdU) incorporation, the DNA synthesis in proliferating cells was determined. BrdU assays were conducted at 24 and 48 h after glioma cells were transfected with siRNA-XIST. Cells were seeded in 96-well culture plates at a density of 2 × 10^3^ cells/well, cultured for 24 or 48 h, then incubated with a final concentration of 10 μM BrdU (BD Pharmingen, San Diego, CA, U.S.A.) for 2 h. When the incubation period ended, the medium was removed, the cells were fixed for 30 min at RT, incubated with peroxidase-coupled anti-BrdU antibody (Sigma–Aldrich) for 60 min at RT, washed three times with PBS, incubated with peroxidase substrate (tetramethylbenzidine) for 30 min, and the 450-nm absorbance values were measured for each well. Background BrdU immunofluorescence was determined in cells not exposed to BrdU but stained with the BrdU antibody.

### Ethical approval

All procedures performed in studies involving human participants were in accordance with the ethical standards of the institutional and/or national research committee and with the 1964 Helsinki declaration and its later amendments or comparable ethical standards.

### Statistics analysis

Data from three independent experiments were presented as mean ± S.D., processed using SPSS 17.0 statistical software (SPSS, U.S.A.). Paired Student’s *t* test was used to compare the expression of *miR-29c* and XIST in glioma tissues and normal tissues. *P*-values of <0.05 were considered statistically significant.

## Results

### Expression of XIST in glioma tissues and its relationship with the clinical features in patients with glioma

In order to investigate the function of XIST in glioma, we first evaluated the expression of XIST in 69 paired glioma tissues and PTBE tissues using real-time PCR assays. The results showed that XIST expression was up-regulated in glioma tissues, compared with that of the PTBE tissues (Figure 1A). In 33.33% (23/69) glioma tissues, XIST had a fold-change of more than 2 compared with the PTBE tissues (Figure 1B). We then divided these samples into two groups according to XIST expression: a high XIST expression group (above the median XIST expression, *n*=35) and a low XIST expression group (below the median XIST expression, *n*=34) (Table 1). As shown in Table 1, lower XIST expression was observed more frequently in patients with advanced WHO stage (III + IV) (*P*<0.001) and larger tumor size (≥5, *P*=0.003). The survival and pathologic features of 69 patients were analyzed using the COX risk proportional regression model. Univariate analysis showed that WHO stage and XIST expression caused significant differences in survival time; multivariate analysis showed that high XIST expression was of high risk (HR =2.037, 95% CI =1.083–3.831) (Table 2). The survival time of patients with glioma with high expression of XIST was shorter than that in patients with low expression of XIST (*P*=0.0007, Figure 1C). We also monitored the expression levels of XIST in all five glioma cell lines, and the results showed that XIST expression was up-regulated in all the five glioma cell lines, U251, U373, LN229, U118, and LN229. The expression of XIST was higher in U251 and LN229 cells than in the other three cell lines (Figure 1D); therefore, U251 and LN229 cell lines were selected as further cell models.

**Figure 1:** Expression of XIST in glioma tissues and its relationship with the clinical features in patients with glioma (**A,B**) Expression of XIST in 69 paired glioma tissues and PTBE tissues were determined using real-time PCR assays. Fold changes of XIST expression was exhibited as log_2_ (tumor/normal). (**C**) Kaplan–Meier overall survival curves for 69 patients with glioma classified according to relative XIST expression level. (**D**) The expression levels of XIST in five glioma cell lines, U251, U373, LN229, U118, LV229, and a normal cell line, NHA, were determined using real-time PCR. The data are presented as mean ± S.D. of three independent experiments; **P<0.01.

### Effects of XIST on glioma cell proliferation and chemoresistance to TMZ

U251 and LN229 cells were transfected with si-XIST to achieve XIST knockdown, as verified using real-time PCR assays (Figure 2A). Cell viability of si-XIST-transfected U251 and LN229 cells was determined using MTT assays. The results showed that XIST knockdown significantly suppressed the cell viability in U251 and LN229 cells (Figure 2B,C). Further, the DNA synthesis capability was also evaluated using BrdU assays. Similar to MTT assays, the DNA synthesis capability was significantly suppressed by XIST knockdown (Figure 2D). These data further demonstrate the role of XIST in promoting glioma cell proliferation. We then investigated whether XIST affects the chemoresistance of glioma cells to TMZ.

**Figure 2:** Effects of XIST on glioma cell proliferation and chemoresistance to TMZ (**A**) siRNA-NC/siRNA-XIST was transfected into LN229 and U251 cells. The expression of XIST was verified using real-time PCR assays. (**B,C**) After transfection with the indicated vectors, the cell viability of LN229 and U251 cells was determined using MTT assays. (**D**) After transfection with the indicated vectors, the cell proliferation of LN229 and U251 cells was determined using BrdU assays. (**E,F**) LN229 and U251 cells were transfected with the indicated vectors. Twenty four hours post-transfection, cells were treated with a series dose of TMZ (0, 30, 60, 120, 240 μM) for 24 h. The cell viability was determined using MTT assays, and the data were presented as a percentage normalized to the viability of cells with 0 μM TMZ treatment. The data are presented as mean ± S.D. of three independent experiments; *P<0.05, **P<0.01. (**G,H**) LN229, TMZ-resistant LN229 (LN229/TMZ), U251, TMZ-resistant U251 (U251/TMZ) cells were treated with a series dose of TMZ (7.5, 15, 30, 60, 120, 240, and 480 μM) for 24 h, and the cell viability of the indicated cells was determined using MTT assays. Data were displayed as a percentage normalized to the viability of cells with no TMZ treatment. The abscissa was the logarithm of TMZ concentration (log-conc.). LC50 represented the concentration of TMZ when cell viability was reduced to 50%. (**I,J**) LN229/TMZ and U251/TMZ cells were transfected with siRNA-NC/siRNA-XIST. Twenty four hours after transfection, cells were treated with a series dose of TMZ (7.5, 15, 30, 60, 120, 240, and 480 μM) for another 24 h; the cell viability was then determined using MTT assays.

Si-XIST-transfected U251 and LN229 cells were treated with a series of concentrations of TMZ (0, 30, 60, 120, 240 μM); and then cell viability was evaluated using MTT assays. The results showed that glioma cell viability was repressed by TMZ treatment in a dose-dependent manner; TMZ-induced repression of glioma cell viability could be amplified by XIST knockdown (Figure 2E,F). These data suggest that XIST is involved in regulation of glioma cell proliferation either in the presence or absence of TMZ; in addition, XIST may affect the chemoresistance of glioma cells to TMZ.

We validated that XIST knockdown can enhance the repressive effect of TMZ on glioma cell proliferation; we then examined the effect of XIST on regulating the chemosensitivity of glioma cells to TMZ. LN229, LN229/TMZ, U251, and U251/TMZ cells were treated with a series of doses of TMZ (7.5, 15, 30, 60, 120, 240, and 480 μM) for 24 h and then monitored for cell viability. The cell viability of untreated cells was defined as 100%. The results showed that for U251 cells, the TMZ concentration to reduce cell viability to 50% was approximately 58.16 μM (lC_50_ =58.16); for U251/TMZ cells this value was 157.2 μM (lC_50_ =157.2) (Figure 2G). Similar results were observed for LN229 cells, the TMZ concentration to reduce LN229 cell viability to 50% was approximately 54.57 μM (lC_50_ =54.57), for LN229/TMZ cells 155.8 μM (lC_50_ =155.8) (Figure 2H). We transfected LN229/TMZ and U251/TMZ cells with siRNA-NC/siRNA-XIST, and then repeated the above assays to validate the effect of XIST on glioma cells’ chemosensitivity. Results showed that XIST knockdown amplified TMZ-induced repression of glioma cells viability and reduced the lC_50_ values to 103.4 (LN229/TMZ) and 99.88 (U251/TMZ) (Figure 2I,J). These data suggested that XIST may exacerbate the chemoresistance of glioma cells to TMZ-based chemotherapy. However, the mechanism by which XIST regulates the chemoresistance of glioma cells to TMZ remains to be investigated.

### XIST regulated *miR-29c* by directly targetting in TMZ-resistant glioma cells

In view of the key role of *miR-29c* in cancers, in particular the chemosensitivity of cancer cells [16,17]; we further investigated whether XIST regulates the chemoresistance of glioma cell to TMZ through *miR-29c*. Mimics NC/*miR-29c* mimics or inhibitor NC/*miR-29c* inhibitor was transfected into LN229/TMZ and U251/TMZ cells to achieve *miR-29c* overexpression or inhibition, and the transfection efficiency was verified using real-time PCR (Figure 3A). The expression of XIST in these cells was monitored using real-time PCR. The results showed that XIST expression was up-regulated by *miR-29c* inhibition while down-regulated by ectopic *miR-29c* (Figure 3B). Then the expression of *miR-29c* in response to XIST knockdown was monitored in LN229/TMZ and U251/TMZ cells. The results showed that *miR-29c* expression was also negatively regulated by XIST (Figure 3C). To investigate the mechanism by which XIST and *miR-29c* regulates each other, we further performed RIP assay to verify the direct binding of *miR-29c* and XIST. RIP results showed that miR-29c and XIST were associated with the AGO2 in LN229/TMZ and U25/TMZ cells (Figure 3D). In RNA extracted from precipitated AGO2 protein, *miR-29c* levels were 3.5 times higher than IgG, and XIST levels were more than two times higher than IgG (Figure 3E). To confirm the interaction between XIST and *miR-29c*, a wt-XIST luciferase reporter gene vector, as well as a mut-XIST luciferase reporter gene vector containing a 5-bp mutation at the putative binding site of *miR-29c* was constructed (Figure 3F). The indicated vectors were cotransfected into TMZ-resistant glioma cell line U251/TMZ with mimics NC/*miR-29c* mimics or inhibitor NC/*miR-29c* inhibitor, and the luciferase activity was then monitored using dual luciferase assays. Results showed that the luciferase activity of the wt-XIST luciferase reporter vector was notably suppressed in response to *miR-29c* mimics transfection while amplified in response to miR-29c inhibitor transfection, compared with control groups (Figure 3G). Additionally, the effect of *miR-29c* mimics or inhibitor on luciferase activity was offset by mutations in XIST (Figure 3G). These data suggest that XIST directly binds to *miR-29c* to inhibit its expression, thereby affecting the chemoresistance of glioma cells to TMZ.

**Figure 3:** XIST regulated *miR-29c* by directly targetting in TMZ-resistant glioma cells (**A**) LN229/TMZ and U251/TMZ cells were transfected with mimics NC/*miR-29c* mimics or inhibitor NC/*miR-29c* inhibitor. Expression of *miR-29c* was verified using real-time PCR assays. (**B**) LN229/TMZ and U251/TMZ cells were transfected with mimics NC/*miR-29c* mimics or inhibitor NC/miR-29c inhibitor. Expression of XIST in response to miR-29c overexpression or inhibition was determined using real-time PCR assays. (**C**) LN229/TMZ and U251/TMZ cells were transfected with siRNA-NC/siRNA-XIST. Expression of *miR-29c* in response to XIST knockdown was determined using real-time PCR assays. (**D,E**) Association of *miR-29c* and XIST with AGO2 in LN229/TMZ and U251/TMZ cells. Detection of AGO2 and IgG using Western blotting (D). Detection of miR-29c and XIST using real-time PCR (E). (**F**) wt-XIST and mut-XIST luciferase reporter gene vectors were constructed by mutating the putative binding site of *miR-29c* in XIST. (**G**) The indicated vectors were cotransfected into the TMZ-resistant glioma cells (U251/TMZ) with *miR-29c* mimics or *miR-29c* inhibitor. The luciferase activity in each group was then determined using dual luciferase assays. The data are presented as mean ± S.D. of three independent experiments; **P<0.01.

### XIST/*miR-29c* axis regulated glioma cell chemoresistance to TMZ through DNA mismatch repair pathway

After confirming that XIST directly binds to *miR-29c* to regulate its expression, next, we assessed the combined effect of XIST and *miR-29c* on glioma cell proliferation and chemoresistance to TMZ. TMZ-resistant U251/TMZ and LN229/TMZ cells were cotransfected with si-XIST and *miR-29c* inhibitor. The cell proliferation of U251/TMZ and LN229/TMZ cells was significantly suppressed by XIST knockdown, whereas promoted by *miR-29c* inhibition; the suppressive effect of XIST knockdown on glioma cell proliferation coule be partially reversed by *miR-29c* inhibition (Figure 4A,B). Furthermore, 24 h after transfection, cells were treated with a series dose of TMZ (7.5, 15, 30, 60, 120, 240, and 480 μM) for 24 h; the cell viability was then determined using MTT assays to assess the combined effect of XIST and *miR-29c* on glioma cell chemoresistance to TMZ. Data were displayed as described; the TMZ concentration to reduce cell viability to 50% (lC_50_) for U251/TMZ and LN229/TMZ was significantly reduced by XIST knockdown, whereas increased by *miR-29c*, indicating that XIST knockdown reduced the chemoresistance of glioma cell to TMZ whereas *miR-29c* inhibition played an opposite role. Moreover, the effect of XIST knockdown on glioma cell chemoresistance could be partially reversed by *miR-29c* inhibition (Figure 4C,D).

**Figure 4:** XIST/*miR-29c* axis regulated glioma cell chemoresistance to TMZ through DNA mismatch repair (MMR) pathway U251/TMZ and LV229/TMZ cells were cotransfected with si-XIST and *miR-29c* inhibitor. (**A,B**) The cell viability and DNA synthesis capability were determined using MTT and BrdU assays. (**C,D**) Twenty four hours after transfection, cells were treated with a series dose of TMZ (7.5, 15, 30, 60, 120, 240, and 480 μM) for 24 h; the cell viability was then determined using MTT assays. Data were displayed as described. (**E**) The protein levels of MSH6 were determined using Western blot assays. (**F**) The protein levels of SP1 and MGMT were determined using Western blot assays. The data are presented as mean ± S.D. of three independent experiments; *P<0.05, **P<0.01. #*P*<0.05, ##*P*<0.01, compared to si-XIST + inhibitor-NC group.

**Figure 5:** The expression levels and correlations of *miR-29c*, SP1, and MGMT in tumor and PTBE tissues (**A**–**C**) Expression of *miR-29c*, SP1, and MGMT mRNA in 69 paired glioma tissues and PTBE tissues was determined using real-time PCR assays. The data are presented as mean ± S.D. of three independent experiments; **P<0.01. (**D**–**F**) The correlation between XIST and *miR-29c, SP1*, and *MGMT* mRNA expression, respectively, was analyzed using Spearman’s rank correlation analysis.

TMZ is one of the most widely used alkylating agents, which modify DNA in several positions, one of which is O6-methylguanine MeG (O6MeG). This modified guanine preferentially pairs with thymine during DNA replication, triggering a DNA mismatch repair (MMR) pathway that ultimately causes DNA double-strand breaks and induces apoptosis [24–26]. Methylation damage can be reversed by MGMT [26]. In addition, SP1 has been reported to regulate one of the key MMR proteins, MSH6 [27]. Here, we investigated whether the MMR pathway were involved in XIST/*miR-29c* regulation of glioma cell chemoresistance to TMZ by measuring the protein levels of MSH6, MGMT, and SP1. MSH6, SP1, and MGMT protein levels were significantly reduced by XIST knockdown, whereas increased by miR-29c inhibition; the suppressive effects of XIST knockdown on the indicated proteins could be significantly reversed by *miR-29c* inhibition (Figure 4E,F). These data indicate that the MMR pathway is involved in XIST/*miR-29c* regulation of glioma cell chemoresistance to TMZ.

### The expression levels and correlations of *miR-29c*, SP1, and MGMT in tumor and PTBE tissues

Finally, to further confirm the above findings, the expression of *miR-29c*, SP1, and MGMT in glioma tissues and the PTBE tissues was monitored using real-time PCR assays. The results showed that in tumor tissues, *miR-29c* expression was down-regulated while SP1 and MGMT mRNA expression was up-regulated as compared with in PTBE tissues (Figure 5A-C). Spearman’s rank correlation coefficient was performed to analyze the correlation between XIST and *miR-29c*, between XIST and PS1, between XIST and MGMT. The results showed that XIST was inversely correlated with *miR-29c*, positively correlated with PS1, positively related with MGMT (Figure 5D-F). Taken together, these data suggest that XIST can inhibit *miR-29c* expression by directly binding to *miR-29c* and subsequently up-regulate the expression of SP1 and MGMT to promote the chemoresistance of glioma cells to TMZ.

## Discussion

TMZ-based chemotherapy is the most commonly used treatment for glioma; however, due to the acquisition of chemoresistance of glioma cells to TMZ, the efficacy is very limited [1,3,28]. Although changes in a number of genetic factors, such as PTEN, VEGF, and EGFR, are associated with the pathogenesis of glioma and the chemoresistance of glioma cells to TMZ [3,29,30], the molecular biology of chemoresistance of glioma cells to TMZ is still largely unknown.

Studies have demonstrated that approximately 18% of these ncRNAs are associated with human tumors, compared with only 9% of human protein-coding genes [31], suggesting that lncRNA can act as a major contributor to carcinogenesis and cancer progression. Moreover, the role of dysregulated lncRNAs in the chemoresistance of many cancers have garnered increased scientific interest in recent years. Accumulating evidence confirms that lncRNAs can affect the sensitivity of cancer cells to chemotherapy. For example, a well-characterized lncRNA, HOTAIR, contributes to the chemoresistance of lung adenocarcinoma and glioma via inhibiting p21 expression [32,33]. Another lncRNA, UCA1, enhances 5-fluorouracil resistance of colorectal cancer by inhibiting *miR-204-5p* [34]. Low XIST expression predicts drug response in PDXs associated with a significant reduction in the breast cancer stem cells population [17]. In the present study, we first evaluated the expression of XIST and its relationship with the clinical features in patient with glioma. XIST expression was significantly up-regulated in glioma tissues and cell lines, compared with PTBE tissues and NHA cell line, respectively; further, a higher XIST expression was correlated with a poorer prognosis in patients with glioma, including larger tumor size, advanced WHO stages, and shorter OS. XIST knockdown significantly suppressed glioma cell proliferation in the presence or absence of TMZ treatment. Upon TMZ treatment, XIST acted on glioma cell proliferation in a dose-dependent manner, indicating the potential role of XIST in regulating the chemoresistance of glioma cell to TMZ.

We then conducted a series of doses of TMZ treatment on non-TMZ-resistant and TMZ-resistant glioma cell lines (U251, U251/TMZ, LN229, and LN229/TMZ). The cell viability of non-TMZ-resistant glioma cells was significantly suppressed by TMZ treatment in a dose-dependent manner; however, the suppressive effects of TMZ on TMZ-resistant glioma cells were attenuated. Then, XIST knockdown was conducted to investigate its role in glioma chemoresistance to TMZ. XIST knockdown reduced the lC_50_ values of both LN229/TMZ and U251/TMZ cells, indicating that XIST aggregated the chemoresistance of glioma cell to TMZ. However, the mechanism by which XIST affects the chemoresistance of glioma cells remains to be investigated.

It has been recently discovered that the interaction between lncRNAs and miRNAs affects post-transcriptional regulation by inhibiting the available miRNA activity. According to previous studies, lncRNA can act as a specific ‘sponge’ for miRNAs to attenuate their regulatory effect on mRNAs [22]. In view of the important role of *miR-29c* in regulating cancer cell growth and invasion [18–20], as well as glioma chemoresistance to TMZ [35], we validated whether XIST affects the chemoresistance of glioma cells to TMZ through *miR-29c*. As shown by real-time PCR, XIST can reduce the detectable amount of *miR-29c*, while up-regulating *miR-29c* expression could reduce XIST expression, indicating that XIST exerted similar regulatory behaviors as *miR-29c* inhibitor, so we speculated that XIST might regulate *miR-29c* expression via the RNAi pathway at the post-transcriptional level. This would suggest that both *miR-29c* and XIST exist in the RISC. Since AGO2 is a key component of the RISC, we therefore performed RIP with the AGO2 antibody. In RNA extracted from precipitated AGO2 protein, we could detect both *miR-29c* and XIST with a more than 2–3.5-fold enrichment compared with IgG. These indicate that *miR-29c* and XIST are associated with each other in glioma cells. To further confirm the interaction between XIST and *miR-29c*, luciferase assays were performed. Consistent with RIP results, XIST interacted with *miR-29c* through direct binding to *miR-29c*, thereby degrading *miR-29c* most possibly through the RISC it carried. Furthermore, we also assessed the combined effect of XIST and *miR-29c* on glioma cell proliferation and chemoresistance to TMZ. XIST knockdown caused significant suppression of glioma cell proliferation and chemoresistance, whereas *miR-29c* inhibition promoted glioma cell proliferation and chemoresistance; the effect of XIST knockdown on the indicated TMZ-resistant glioma cells could be partially reversed by *miR-29c* inhibition. These data suggest that XIST can directly bind to *miR-29c* to inhibit its expression, thereby affecting glioma cell proliferation and chemoresistance to TMZ.

TMZ is the most widely used alkylating agent that modifies DNA at several positions, one of which is O6MeG. This modified guanine preferentially pairs with thymine during DNA replication which initiates the MMR pathway, and then ultimately causes DNA double-strand break and induces apoptosis [24–26]. The methylation damage can be reversed by MGMT [26]. Although various mechanisms that mediate the intrinsic or acquired resistance of TMZ have been recognized, MGMT is now considered to play a major role in mediating the resistance of TMZ and other alkylating agents [36]. The intracellular levels of the alkylating enzyme MGMT interfere with TMZ response in patients with glioblastoma multiform [37,38]. In addition to MGMT, SP1 has been reported to regulate a key MMR protein MSH6 [27] by affecting the promoter activity of MSH6. In the present study, we monitored the protein levels of MSH6, MGMT, and SP1 in response to cotransfecting XIST and* miR-29c* in TMZ-resistant glioma cell lines. XIST knockdown significantly reduced MSH6, SP1, and MGMT proteins, whereas miR-29c inhibition significantly increased MSH6, SP1, and MGMT proteins; the suppressive effect of XIST knockdown on these proteins could be partially reversed by *miR-29c* inhibition. These data suggest that XIST/*miR-29c* may modulate the chemoresistance of glioma cells to TMZ by modulating the MMR pathway.

In the glioma tissues, *miR-29c* expression was down-regulated, whereas SP1 and MGMT mRNA expression was up-regulated; moreover, XIST was inversely correlated with *miR-29c*, whereas positively correlated with SP1 and MGMT expression in glioma tissues, indicating that targetting XIST to rescue *miR-29c* expression, thereby inhibiting the chemoresistance of glioma cells to TMZ may be a promising strategy for improving the efficiency of TMZ-based chemotherapy.

## Abbreviations

AGO2: argonaute 2
BrdU: 5-bromo-2-deoxyuridine
CI: confidence interval
COX: Cox's proportional hazards regression model
CSU: Central South University
Ct: comparative cycle threshold
EGFR: epidermal growth factor receptor
GAPDH: glyceraldehyde-3-phosphate dehydrogenase
HOTAIR: HOX transcriptional antisense RNA
HR: hazard ratio
HRP: horseradish peroxidase
lncRNA: long non-coding RNA
MGMT: O^6^-methylguanine-DNA methytransferase
MMR: mismatch repair
MSH6: mutS homolog 6
mut: mutant-type
ncRNA: non-coding RNA
NHA: normal human astrocyte
OD_490 nm_: optical density at a wavelength of 490 nm
O6MeG: O^6^-methylguanine MeG
OS: overall survival
PDX: patient-derived xenograft
PTBE: peritumoral brain edema
PTEN: phosphatase and tensin homolog deleted on chromosome ten
qRT-PCR: quantitative real-time polymerase chain reaction
RIP: RNA immunoprecipitation
RISC: RNA-induced silencing complex
RIPA: radio-immunoprecipitation assay
RPMI-1640: Roswell Park Memorial Institute 1640
RT: room temperature
si-XIST: siRNA for XIST
SP1: specificity protein 1
TMZ: temozolomide
VEGF: vascular endothelial growth factor
wt: wild-type
XIST: X inactive specific transcript
